The article "Expression Profile of MAGE-B1 Gene and Its Hypomethylation Activation in Colon Cancer" was retracted in 2024. Reasons: signs of a paper mill; suspected computer-generated content; unreliable results or conclusions; concerns about the data.

# Expression Profile of MAGE-B1 Gene and Its Hypomethylation Activation in Colon Cancer

**DOI:** 10.1155/2022/6066567

**Published:** 2022-07-27

**Authors:** Mikhlid H. Almutairi, Mona M. Alotaibi, Rasha Alonaizan, Bader O. Almutairi

**Affiliations:** Zoology Department, College of Science, King Saud University, P.O. Box: 2455, 11451 Riyadh, Saudi Arabia

## Abstract

Cancer-testis (CT) genes are typically expressed in the testes; however, they have been linked to aberrant expression in a variety of malignancies. *MAGE-B* family genes are an example of CT genes. Therefore, the overarching objective of this study was to examine the expressions of *MAGE-B* family genes in several patients with colon cancer (CC) to see if they might be employed as cancer biomarkers in the early phases of cancer detection and to improve treatment. In this investigation, RT-PCR was used to analyze *MAGE-B* family genes in neighboring normal colon (NC) tissue from 10 CC patients. In addition, the effect of DNA demethylation on the expression status of the *MAGE-B1* gene was evaluated by RT-PCR in HCT116 and Caco-2 cells and by qRT-PCR for HCT116 only after treating both CC cell lines with varying concentrations of 5-aza-2′-deoxycytidine (1.0, 5.0, and 10.0 *μ*M) for 48 or 72 hours. All *MAGE-B* family genes except for *MAGE-B1* showed weak bands in several samples of NC tissues: *MAGE-B2*, *MAGE-B3*, *MAGE-B4*, *MAGE-B5*, and *MAGE-B6* genes were observed in 40%, 50%, 40%, 30%, and 60% of the NC samples, respectively. Nonetheless, they had strong bands in multiple samples of CC tissues, with 70%, 90%, 60%, 50%, and 90% of the CC samples, respectively. Interestingly, *MAGE-B1* was detected in 60% of CC tissues but not in NC tissues, suggesting that it is a potential biomarker for early CC detection. *MAGE-B1* expression was not observed in either untreated or DMSO-treated HCT116 cells after 48 or 72 hours of treatment. However, according to the RT-PCR and qRT-PCR results, the *MAGE-B1* gene was overexpressed in the HCT116 cells treated with three different concentrations of 5-aza-2′-deoxycytidine. This shows that demethylation plays a crucial role in *MAGE-B1* expression activation.

## 1. Introduction

Colon cancer (CC) is a leading cause of mortality globally, and its incidence is anticipated to double by 2030 [1]. Between nations, CC incidence and death rates vary around tenfold, with the highest rates reported in wealthy countries, where they have remained relatively stable. However, rates are rapidly increasing in developing nations [1]; despite the fact that CC screening programs have reduced incidence rates around the globe, mortality rates continue to rise in certain locations [2, 3]. In Saudi Arabia, CC is the most prevalent type of cancer in men and the third most common in women [4–6]. The majority of CC instances in Saudi Arabia are detected during clinical exams rather than through screening initiatives. Screening for CC can help reduce the incidence of death and mortality associated with this condition, as CC is a slow-progressing disease that can be treated if detected early. Therefore, the development of a noninvasive biomarker for early disease detection could be advantageous [7]. CC carcinogenesis is a multistep process involving oncogene and tumor suppressor gene alterations that results in the gradual transformation of the normal colorectal epithelium into adenoma, invasive tumor, and metastatic tumor [8]. CC has been associated with a variety of risk variables, including ethnic origin, environment, and genetics [9].

The article "Expression Profile of MAGE-B1 Gene and Its Hypomethylation Activation in Colon Cancer" was retracted in 2024. Reasons: signs of a paper mill; suspected computer-generated content; unreliable results or conclusions; concerns about the data.

Early identification and successful cancer therapy continue to be substantial clinical hurdles. Thus, there is an urgent need to identify novel tumor-associated chemicals that can be exploited to develop novel clinical diagnostics and therapeutic targets for a variety of cancers [10]. Numerous studies on diverse antigen classes as potential novel cancer-specific biomarkers for early detection of malignancy have been conducted. Cancer-testis (CT) antigens are a type of cancer-specific antigen that express proteins only in human germ line cells of the testis and cancer cells [11]. Due to their particular, cancer-specific expression pattern, CT antigens could be useful as cancer biomarkers and treatments [11, 12].

CT expression is seen in a variety of tumor types, including ovarian, colon, and melanoma [13]. In cancer tissue, aberrant expression of these CTs could play a critical role in tumor growth, proliferation, and antiapoptotic processes [14]. van der Bruggen et al. discovered the first CT gene in a patient with malignant melanoma and designated it a part of the melanoma antigen family (MAGE-1) [15]. Most CT genes are situated on the X chromosome [16]; are classified as member of multicopy, paralogous gene families; and express splice variants, including the *MAGE-A*, *GAGE*, *PAGE*, *XAGE1*, and *SSX* families.

MAGEs are encoded by a paralogous gene family consisting of about 60 genes [17]. Although their function in testis germ cells is unknown, their oncogenic activity is widely documented [18]. The first member of the human MAGE family that was identified is a member of a cluster of 12 MAGE-A genes found on the Xq28 [19]. Following that, a second cluster, dubbed MAGE-B, was discovered in human Xp21 [20], and, lastly, another cluster, dubbed MAGE-C, was located in Xq26–27 [21]. They are completely inactive in normal tissues, as they are a component of male germ cells. Unexpectedly, MAGEs have been found to be frequently expressed in a range of cancers [22], including colorectal, melanoma, breast, and esophageal [22–25].

The article "Expression Profile of MAGE-B1 Gene and Its Hypomethylation Activation in Colon Cancer" was retracted in 2024. Reasons: signs of a paper mill; suspected computer-generated content; unreliable results or conclusions; concerns about the data.

The MAGE-B family, including MAGE-B1, MAGE-B2, MAGE-B3, and MAGE-B4 genes, is strongly homologous with the MAGE-A gene family. *MAGE-B* gene expression was not detected in normal tissues except the testis. However, *MAGE-B1* and *MAGE-B2* genes were significantly expressed among various types of cancer, such as esophageal, gastric, and colorectal carcinoma [25]. *MAGE-B2* and *MAGE-B3* genes were overexpressed in hepatocellular carcinoma and colorectal cancer patients [22, 26]. Additionally, they are often exhibited in cancer patients from a variety of ethnic backgrounds, including German, Chinese, Taiwanese, Italian, and Japanese [22, 25–28].

DNA methylation regulates the expression of numerous CT genes and is mostly carried out in the gene promoter region by DNA methyltransferase enzymes (DNMTs) [29]. The expression of certain CT genes, such as *MAGE-A1* in oral carcinoma and *MAGE-A4* in thyroid cancer, is apparently enhanced by DNA hypomethylation [30, 31]. Treatment of colon and ovarian cancer cell lines with a DNA methyltransferase 1 inhibitor (DNMTi), 5-aza-2′-deoxycytidine, can stimulate the expression of many CT genes [32, 33].

The expression patterns of *MAGE-B* family genes have not been examined in Saudi populations with CC. Thus, the overall purpose of this study was to analyze the expression of *MAGE-B* genes in Saudi patients with CC to identify potential cancer biomarkers that might aid in the early identification and treatment of CC.

## 2. Materials and Methods

### 2.1. Collecting Samples and Obtaining Ethical Approval

In this study, CC and normal colon (NC) tissues were taken from 10 Saudi male patients who had not received any treatment, including chemotherapy, physiotherapy, or radiation. Stabilization solution for *RNAlater* was stored in an Eppendorf tube (Thermo Fisher Scientific; 76106). Ethical approval was provided by the Al-Imam Muhammad Ibn Saud Islamic University with IRB number HAPO-01-R-011 and project number 214/2022 [34]. Patients were asked to sign a permission form and complete a survey as well as a self-administered questionnaire that inquired about their age, social behaviors, family history of cancer, and personal medical history.

### 2.2. Primer Design for the Selected Genes

The National Center for Biotechnology Information's (http://www.ncbi.nlm.nih.gov/) database was used to generate primers for each gene. Then, using the Primer-BLAST program (https://www.ncbi.nlm.nih.gov/tools/primer-blast/), individual primers for each gene were constructed. Macrogen Company (Seoul, South Korea) synthesized the designed primers at a final concentration of 10 *μ*M for use in studies (https://dna.macrogen.com). The primer sequences and predicted sizes of each gene are listed in Table 1.

The article "Expression Profile of MAGE-B1 Gene and Its Hypomethylation Activation in Colon Cancer" was retracted in 2024. Reasons: signs of a paper mill; suspected computer-generated content; unreliable results or conclusions; concerns about the data.

### 2.3. Human CC Cell Line, HCT116, and Caco-2: Source and Culture

The HCT116 and Caco-2 cells were obtained from the American Type Culture Collection (ATCC, Manassas, VA, USA), and the cells were cultured in DMEM (Thermo Fisher Scientific; 61965026) supplemented with 10% fetal bovine serum (FBS) (Thermo Fisher Scientific; A3160801) and penicillin-streptomycin (Thermo Fisher Scientific; 15140122) and then kept in the incubator with 5% CO_2_ at 37°C.

### 2.4. 5-Aza-2′-Deoxycytidine Treatment of HCT116 and Caco-2 Cell Lines at Various Concentrations

For 48 or 72 hours, the HCT116 and Caco-2 cell lines were treated with various concentrations of demethylating agent (5-aza-2′-deoxycytidine) 1.0, 5.0, and 10.0 *μ*M, whereas the control cells received the same concentration of drug solvent DMSO. Every 24 hours, the media was refreshed.

### 2.5. Extraction of Total RNA and Production of Complementary DNA (cDNA)

Fifty milligrams of tissues and about 3 × 10^6^ cells of cultivated cells were used to extract the total RNA using the All Prep DNA/RNA Mini Kit (Qiagen; 80204), according to the manufacturer's guidelines. The Nano-Drop8000 spectrophotometer was then used to determine the RNA concertation. To convert 1 *μ*g of RNA to cDNA, the High-Capacity cDNA Reverse Transcription Kit (Applied Biosystems; 4368814) was used, according to the manufacturer's instructions. After dilution to a 1 : 10 concentration, the cDNA was kept at –20°C until needed.

### 2.6. RT-PCR with Gel Electrophoresis

The PCR reaction, which comprised 100 ng of cDNA, 0.25 *μ*M of reverse and forward primers, and 1X of BioMix Red (BioLine; BIO-25006), was left in the PCR machine for 5 minutes, followed by 35 cycles at 96°C for 30 seconds, 58°C for 30 seconds, and 72°C for 30 seconds, respectively. The run was concluded with a 5-minute warm-up at 72°C. Finally, the PCR results were examined in a 1% agarose gel containing 0.5 g/mL of ethidium bromide. A total of 3 *μ*L of 100 bp DNA marker (New England Biolabs; N0467) was added to determine the size of the PCR result.

### 2.7. Purification and Sequencing of RT-PCR Products

15 *μ*L of cDNA (15 ng/*μ*L) and 20 *μ*L of forward and/or reverse primers (5 pmol/*μ*L) were inserted into two clean, separate Eppendorf tubes (1.5 mL). Then, the Microgen Company received both tubes for DNA sequencing. The resultant sequencing of each product was uploaded to the BLAST website (https://blast.ncbi.nlm.nih.gov/Blast.cgi) for comparison with the NCBI database.

The article "Expression Profile of MAGE-B1 Gene and Its Hypomethylation Activation in Colon Cancer" was retracted in 2024. Reasons: signs of a paper mill; suspected computer-generated content; unreliable results or conclusions; concerns about the data.

### 2.8. Real-Time Quantitative Polymerase Chain Reaction (qRT-PCR) Primer Design

All primers were designed manually and had an amplicon size below 175 bp to facilitate qRT-PCR amplification. Each primer was 20 nucleotides in length and included 50% G/C to prevent the internal secondary structure that was expected. To avoid the creation of primer dimers, the forward and reverse primers lacked significant complementarity at their 3′ ends and melted at the same temperature. To guarantee primer specificity, a BLAST search was performed on them. Commercially available primers were produced (Macrogen Inc., South Korea), and their sequences are presented in Table 2. The stock primers were diluted to a final concentration of 10 pmol using sterile distilled water.

### 2.9. The qRT-PCR Setup

The qRT-PCR tests were performed according to the manufacturer's instructions using the iTaq Universal SYBR Green Supermix (Bio-Rad; 1725120, Hercules, CA, USA). The volume was then adjusted to 10 *μ*L on a 96-well plate by adding 5 *μ*L of SYBR Green Supermix, 2 *μ*L of cDNA (200 ng), 0.25 *μ*L of each primer, and lastly water. Three duplicate samples were amplified utilizing a 30-second predenaturation step at 95°C, followed by 40 cycles of 15-second denaturation at 95°C, 30-second primer annealing at 58°C, and 15-second extension at 95°C. Following the completion of the 40 cycles, a melting curve study was conducted. *GAPDH* was utilized as a positive control to normalize the qRT-PCR results. qRT-PCR was performed using a QuantStudio 7 Flex Real-time PCR System (Applied Biosystems, Hercules, CA, USA).

### 2.10. Statistical Analyses

Statistical analysis was conducted using SPSS version 22 (SPSS Inc., Chicago, USA). The comparisons between the expressions of *MAGE-B* genes in NC and CC groups and *MAGE-B1* gene in the untreated and treated of HCT116 cell lines were analyzed using an unpaired Student's *t*-test. The findings were provided as average ± SD. All *P* values were statistically significant (^∗^*P* < 0.05 and ^∗∗^*P* < 0.01).

## 3. Results

### 3.1. Clinical Data on the Studied Subjects

Table 3 summarizes the demographic and clinical features of the study participants. The mean age of the 10 CC patients on diagnosis was 57 years (range: 24 to 83 years). Fifty percent of CC patients were under the age of 57, and 50% were over the age of 57.

### 3.2. Expression Profile of *MAGE-B* Genes in CC and Matched Adjacent NC Tissues

In this paper, the expressions of six members of the *MAGE-B* family (*MAGE-B1*, *MAGE-B2*, *MAGE-B3*, *MAGE-B4*, *MAGE-B5*, and *MAGE-B6*) were investigated in different samples of CC and their matching NC samples. The RT-PCR validation process began with the identification of *MAGE-B* family genes in various RNAs extracted from 10 NC tissues to determine their testis specificity. Testis cDNA was synthesized from total RNA of human testis and used to verify the primers for each *MAGE-B* gene (Thermo Fisher Scientific; AM7972). The *ACTB* gene expression was utilized as a positive control to determine that the cDNA was of acceptable quality.

The article "Expression Profile of MAGE-B1 Gene and Its Hypomethylation Activation in Colon Cancer" was retracted in 2024. Reasons: signs of a paper mill; suspected computer-generated content; unreliable results or conclusions; concerns about the data.

In this study, no expression of *MAGE-B1* was detected in NC (Figure 1, left side), whereas 60% of CC displayed its expression (Figure 1, right side). The transcriptional level of *MAGE-B2*, *MAGE-B3*, *MAGE-B4*, *MAGE-B5*, and *MAGE-B6* was faintly seen in 40%, 50%, 40%, 30%, and 60% of NC, respectively (Figure 1, left side). However, 70%, 90%, 60%, 50%, and 90% of CC, respectively, showed strong induction of *MAGE-B2*, *MAGE-B3*, *MAGE-B4*, *MAGE-B5*, and *MAGE-B6* expression consecutively (Figure 1, right side). Furthermore, this study analyzed the positive (the case was designated as positive if a band was found) expressions for genes from *MAGE-B2* to *MAGE-B6* in NC and CC tissues. Only *MAGE-B3* showed a statistically significant positive expression in CC compared with NC tissues (*P* = 0.0543, Table 4). Intriguingly, because *MAGE-B1* was not expressed in any of the matched NC tissues but was expressed in 60% of CC tissues (*P* = 0.0017, Table 4), it might be regarded a potential CT gene marker and could be used for early CC diagnosis. A total of three CC samples selected at random from *MAGE-B1* that had positive findings were sequenced to confirm the RT-PCR results.

### 3.3. Epigenetic Modification of *MAGE-B1* Expression in HCT116 and Caco-2 Cell Lines

The DNA methylation status controls and regulates the expression of many CT genes at the promoter level [29]. Thus, HCT116 and Caco-2 cell lines were subjected to a methylation-modifying agent, 5-aza-2′-deoxycytidine, to investigate the effect of DNA demethylation on the *MAGE-B1* gene expression status. For 48 or 72 hours, three different doses of 5-aza-2′-deoxycytidine (1.0, 5.0, and 10.0 *μ*M) were employed. Because the drug was dissolved in DMSO, both cell lines were treated with DMSO to compare gene expression. Additionally, untreated HCT116 and Caco-2 cells were employed as negative controls to evaluate *MAGE-B1* gene expression in treated and untreated cells. The normal testis was used as a positive control for primer efficacy, whereas the *ACTB* gene was used to determine the quality of cDNA. *SSX2* is a well-characterized CT gene that was utilized as a positive control to assess its expression. The expression of the *MAGE-B1* gene was determined first by RT-PCR and then by qRT-PCR, as shown in Figures 2 and 3.

The article "Expression Profile of MAGE-B1 Gene and Its Hypomethylation Activation in Colon Cancer" was retracted in 2024. Reasons: signs of a paper mill; suspected computer-generated content; unreliable results or conclusions; concerns about the data.

RT-PCR results shows that *MAGE-B1* expression was not observed in untreated or DMSO-treated HCT116 cells after 48 or 72 hours of treatment. However, the band intensities of this gene were significantly greater in HCT116 and Caco-2 cells treated with three different doses of 5-aza-2′-deoxycytidine than in untreated cells after 48 and 72 hours of treatment.

qRT-PCR was also performed to determine whether RT-PCR results correlates with qRT-PCR results for *MAGE-B1* expression in HCT116 cells following treatment with 1.0, 5.0, and 10.0 *μ*M of 5-aza-2′-deoxycytidine. Notably, the expression of *MAGE-B1* was significantly increased after 48 and 72 hours of exposure to the three doses of 5-aza-2′-deoxycytidine in comparison to cells treated with DMSO (Figure 3). The highest expression of *MAGE-B1* mRNA was detected after treating HCT116 cells with 10.0 *μ*M 5-aza-2′-deoxycytidine for 48 and 72 hour. Taken together, these findings indicated that the *MAGE-B1* expression can be upregulated by the demethylating agent.

## 4. Discussion

CC is a leading cause of mortality in Saudi Arabia, affecting predominantly elderly persons. Nonetheless, it now affects people of all ages [6, 35]. As a result, biomarkers for the early stages of CC must be found to reduce death and mortality rates [6, 7]. The MAGE gene produces CT antigens, which are expressed preferentially in a variety of human malignancies but not in normal tissues [36]. However, the *MAGE-B* gene expression profiles in Saudi populations with CC are unclear. As a result, this research sought to obtain a better understanding of the *MAGE-B* gene expression patterns and their epigenetic regulation.

In this study, RT-PCR was used to analyze *MAGE-B* family genes in CC tissues and neighboring NC tissues. Any genes that were expressed in CC tissues but not in NC tissues might serve as a biomarker for early diagnosis and treatment (such as immunotherapy) of CC in the Saudi population. Immunotherapy for cancer has demonstrated long-term outcomes in individuals with advanced illness, which are not observed with the conventional treatment of chemotherapy [37].

In this work, RT-PCR was used to validate *MAGE-B* family genes in various Saudi CC tissues compared with their neighboring NC tissues. For the first time, this paper demonstrated that the *MAGE-B2*, *MAGE-B3*, *MAGE-B4*, *MAGE-B5*, and *MAGE-B6* genes exhibited PCR products that were distinct from those seen in NC tissues. However, the band intensities in CC tissues were stronger than in NC tissues. Additionally, the positive *MAGE-B3* expression in CC tissues was more statistically significant than in NC tissues. This pattern was also found in prior studies on *MAGE-B2* and *MAGE-B3* gene expressions in esophageal cancer cell lines [25] and in Taiwanese patients with colorectal cancer [22], consistent with findings in this study. In comparison, *MAGE-B1* was found as a viable candidate for CC markers in the Saudi population because it was expressed in a variety of 60% CC samples but not in NC samples. However, because the sample size was small in that study, more research is required to elucidate the expression of *MAGE-B* genes in different types of malignancies. In a previous work, a similar result was detected for *MAGE-B1* mRNA in approximately 45% of hepatocellular carcinoma, whereas it was not detected in the neighboring normal liver tissues [26]. This is most likely related to the activation of CT genes in cancer. Demethylation, for example, can result in the activation of previously identified CT genes in cancer [33].

The article "Expression Profile of MAGE-B1 Gene and Its Hypomethylation Activation in Colon Cancer" was retracted in 2024. Reasons: signs of a paper mill; suspected computer-generated content; unreliable results or conclusions; concerns about the data.

In malignancies, the regulatory mechanisms that control expression of *MAGE-B* genes remain unclear. However, DNA methylation has been found to regulate in *MAGE-A* gene expressions [36]. De Smet et al. demonstrated that demethylation of the CpG sites in promoter of *MAGE-A1* gene is correlated with high levels of gene transcription [38]. To determine whether DNA methylation inhibition induces *MAGE-B1* expression, HCT116 cells were treated for 48 or 72 hours with various concentrations of 5-aza-2′-deoxycytidine. In this study, it was demonstrated that 5-aza-2′-deoxycytidine treatment of HCT116 cells induces *MAGE-B1* expression, indicating that DNA methylation plays a role in the regulation of this gene. Although there are no previous studies on the correlation between genetic hypomethylation and *MAGE-B1* expression, these findings will be interesting and are in accordance with those found in other reports on *MAGE-A* family genes [31, 39, 40].

In this study, *MAGE-B1* was identified as a gene biomarker for the early detection of CC, which might help in the screening of potential CC candidates. However, the present study includes weaknesses. First, only ten samples from CC patients were used, and the results must be replicated with larger number of samples. Second, it was unable to determine the protein levels of the putative MAGE-B1 genes in CC due to a shortage of samples.

## 5. Conclusions

The expression patterns of *MAGE-B* family genes in CC and NC tissues were examined to determine whether any *MAGE-B* gene biomarkers might assist in the early detection of the disease. The mRNA expression of the *MAGE-B1* gene was found in 60% of individuals with CC but not in nearby NC tissues. The pattern of expression of this gene in CC samples implies that it might be employed as a biomarker for malignancy. Additional studies at the protein level and with a bigger cohort of patients are required to validate this finding. Furthermore, it was identified that hypomethylation has a fundamental role in activating *MAGE-B1* gene expression. This observation indicates that its expression is upregulated and could play a crucial role in the genesis and progression of CC.

The article "Expression Profile of MAGE-B1 Gene and Its Hypomethylation Activation in Colon Cancer" was retracted in 2024. Reasons: signs of a paper mill; suspected computer-generated content; unreliable results or conclusions; concerns about the data.

## Figures and Tables

**Figure 1:** Expression profile of *MAGE-B* genes in CC and matched adjacent NC tissues. The *MAGE-B1*, *MAGE-B2*, *MAGE-B3*, *MAGE-B4*, *MAGE-B5*, and *MAGE-B6* genes were examined on 1% agarose gels. Total RNA from 10 NC tissues (left side) and 10 CC tissues (right side) was used to make cDNAs. Testis cDNA was used to validate the primers for each gene. As a positive control for the cDNA samples, *ACTB* expression was used. The expected size of each gene's product is indicated on the left between brackets.

**Figure 2:** The effects of 5-aza-2′-deoxycytidine on MAGE-B1 gene expression in the CC cell lines. MAGE-B1 gene expression was exhibited in 1% agarose gels following treatment with a variety of 5-aza-2′-deoxycytidine doses (1.0, 5.0, and 10.0 *μ*M) for 48 h (left side) or 72 hours (right side). Untreated HCT116 and Caco-2 cells were used for comparison with treated cells. Testis cDNA was used to validate the primer efficiency of the MAGE-B1 gene. HCT116 and Caco-2 cells were treated with DMSO as a control, as DMSO was utilized to prepare the 5-aza-2′-deoxycytidine solution. As a positive control for the cDNA samples, ACTB expression was used. The expected size of each gene's product is indicated on the left between brackets.

**Figure 3:** qRT-PCR analysis of *MAGE-B1* expression in the HCT116 cell line. The gene expression data for *MAGE-B1* in the HCT116 cell line is shown in the bar chart. The *GAPDH* reference gene was used to normalize the expression data. The error bars indicate the standard error of the mean for three repeats (^∗^*P* < 0.05 and ^∗∗^*P* < 0.01). *N* denotes the number of samples.

**Table 1:** Primer sequences and their expected product sizes for *ACTB*, *MAGE-B* family, and *SSX2* genes.

Official gene		Primer direction and sequence (from 5′➔3')	Ta	Product size (bp)
Symbol	Full name			
*ACTB*	Actin beta	Forward: AGAAAATCTGGCACCACACC	58	553
		Reverse: AGGAAGGAAGGCTGGAAGAG		
*MAGE-B1*	MAGE family member B1	Forward: CAGGAATGCTGATGCACTTC		524
		Reverse: GAGGACTTTCATCTTGGTGG		
*MAGE-B2*	MAGE family member B2	Forward: CACTGAAGCAGAGGAAGAAG		467
		Reverse: GGTCTACCTTGTCGATGAAG		
*MAGE-B3*	MAGE family member B3	Forward: GACTCCTATGTCCTTGTCAG		464
		Reverse: GCACTACTGCCATCATTGAG		
*MAGE-B4*	MAGE family member B4	Forward: TCTTTGGCCTTGCCTTGAAG		524
		Reverse: GGAATACGCACTAGTCATGG		
*MAGE-B5*	MAGE family member B5	Forward: CAGTAGAGATGAGGAGTACC		472
		Reverse: GGGCTCTCCATAGATGTAGT		
*MAGE-B6*	MAGE family member B6	Forward: GCGCTTAAGCAAAGATGCTG		473
		Reverse: GCCGGTAAACCACGTACTTA		
*SSX2*	SSX family member 2	Forward: CAGAGAAGATCCAAAAGGCC		407
		Reverse: CTCGTGAATCTTCTCAGAGG		

Abbreviations: Ta: temperature of annealing for each gene; bp: base pair.

The article "Expression Profile of MAGE-B1 Gene and Its Hypomethylation Activation in Colon Cancer" was retracted in 2024. Reasons: signs of a paper mill; suspected computer-generated content; unreliable results or conclusions; concerns about the data.

**Table 2:** Primer sequences and their expected product size for qRT-PCR.

Official gene		Primer direction and sequence (from 5′➔3′)	Ta^∗^	Product size
Symbol	Full name			
*GAPDH*	Glyceraldehyde-3-phosphate dehydrogenase	Forward: GGGAAGCTTGTCATCAATGG	58	173 bp
		Reverse: GAGATGATGACCCTTTTGGC		
*MAGE-B1*	MAGE family member B1	Forward: GAAGGCAGATATGCTGAAGG		125 bp
		Reverse: CACTAGGGTTGTCTTCCTTC		

Abbreviations: Ta: temperature of annealing for each gene; bp: base pair.

**Table 3:** Clinical characteristics of the research participants.

Clinical parameters	CC *N* (%)	NC *N* (%)
Participants	10 (100%)	10 (100%)
Mean of age (min-max)	57 (24-83)	
Below 57	5 (50%)	5 (50%)
Above 57	5 (50%)	5 (50%)

Abbreviations: CC: colon cancer; NC: normal colon; *N*: number of samples.

**Table 4:** Positive expression of *MAGE-B* genes in NC and CC tissues.

*MAGE-B* genes	Number of positive expression in NC (%)	Number of positive expression in CC (%)	*P* value
*MAGE-B1*	0 (0)	6 (60)	**0.0017** ^∗∗^
*MAGE-B2*	4 (40)	7 (70)	0.1963
*MAGE-B3*	5 (50)	9 (90)	**0.0543** ^∗^
*MAGE-B4*	4 (40)	6 (60)	0.3978
*MAGE-B5*	3 (30)	5 (50)	0.3880
*MAGE-B6*	6 (60)	9 (90)	0.1345

Abbreviations: NC: normal colon cancer; CC: colon cancer. Note: values in bold represent a significant result as ^∗^*P* < 0.05 and ^∗∗^*P* < 0.01.

## Data Availability

All the data relevant to this study is mentioned in the manuscript. There is no supplementary data.
